# Comparison of Outcomes between Two Surgical Techniques for Patients with Intestinal Neuronal Dysplasia

**DOI:** 10.1155/2022/9165651

**Published:** 2022-07-21

**Authors:** Yu Lin, Dianming Wu, Yong Shen, Yuanbin He, Jianxin Ye

**Affiliations:** ^1^Pediatric Surgery Department, Fujian Maternity and Child Health Hospital, College of Clinical Medicine for Obstetrics & Gynecology and Pediatrics, Fujian Medical University, Fuzhou, 350000 Fujian, China; ^2^Department of Gastrointestinal Surgery 2 Section, The First Hospital Affiliated to Fujian Medical University, Fuzhou, 350000 Fujian, China

## Abstract

**Objective:**

Hirschsprung disease (HSCR) is a serious congenital intestinal disease with a prevalence of 1/5000. HSCR remains one of the most severe congenital malformations of the abdominal organs in children that require complex reconstructive surgery. This study is aimed at investigating the clinical analysis of ileal Santulli stoma and ileal double-lumen stoma in children diagnosed with intestinal neuronal dysplasia (IND).

**Methods:**

Retrospective analysis was performed on the children who were admitted to our hospital for intestinal obstruction from January 2014 to January 2019, underwent fistula operation and fistula closure operation, and were diagnosed with IND. According to the different modes of fistula, the children were divided into ileal Santulli stoma group and ileal double-lumen stoma group. The body weight of the children in the two groups during the second stage of fistula closure operation was compared. The number of hospitalizations due to enteritis and dehydration during the two operations was compared.

**Results:**

A total of 23 cases (12 males and 11 females) were included in this study, including 10 cases in the Santulli group and 13 cases in the ileal double-lumen stoma group. There were no significant differences in baseline data and fistula location between the two groups. Compared with the ileal double-lumen stoma group, the Santulli stoma group had significantly higher weight of fistula precursor (*P* < 0.05), the interval between two operations was shorter (*P* < 0.05), there is less hospitalization for enteritis and dehydration during the two operations (*P* < 0.05), and there is less economic cost after fistula (*P* < 0.05).

**Conclusion:**

The clinical effect of ileum Santulli fistula is significantly better than double-lumen ileum fistula, which is not only beneficial to the growth and development of children after the first fistula but also can shorten the time of fistula closure, reduce the incidence of dehydration, and reduce the economic burden of family members. Therefore, it is worthy of clinical promotion and application.

## 1. The Background

Hirschsprung's disease (HSCR) is a common surgical disease in children. The main cause is the deficiency of ganglion cells in the distal submucosal and intermuscular ganglion of the intestinal canal due to the development of intestinal neurons in the embryonic stage. The main clinical manifestations include delayed meconium discharge, abdominal distention, intractable constipation, and intestinal obstruction [1, 2]. During the operation, there is no obvious appearance of Hirschsprung's colon, such as the stenosis segment, the transitional segment, and the expansion segment, and some of them are characterized by uniform colon stenosis with intestinal wall hyperemia and edema or thick and stiff intestinal wall [3]. In clinical practice, there are sometimes clinical manifestations similar to Hirschsprung's disease, but there are ganglion cells in intestinal biopsy, which are manifested as abnormal development of intestinal ganglion cells, including dysplasia of intestinal neurons, immature intestinal neurons, and reduction of intestinal neurons. Intraoperative frozen rapid section can only determine the presence or absence of ganglion cells and is not yet able to make an accurate diagnosis of complex neuropathy such as abnormal development of intestinal neurons. Multisite full-thickness colorectal biopsy is a reliable means to confirm HAD [4–6]. Some of these children can present with progressive abdominal distention, vomiting, and constipation within three months of birth, which can lead to failure to feed in serious cases and even intestinal obstruction, intestinal necrosis, and perforation, requiring emergency surgery [7]. The clinical treatment of such children is difficult.

Internal rectal pull through (ERP) and Duhamel pull through are the most common final operations for HSCR [8, 9]. Both ERP and Duhamel can be performed laparoscopy- or laparotomy-assisted, although ERP can also be performed entirely transanally in rectosigmoid HSCR [10, 11]. However, due to the distal intestinal neuronal dysplasia lesions early intestinal canal length and function cannot clear, ileostomy is often required. In the past, double-lumen ileum fistula was often performed in our department, which can significantly improve symptoms such as abdominal distention, constipation, and intestinal obstruction. However, poor weight gain, dehydration, and long interval between secondary fistula closure and high economic costs often occurred after surgery.

Ileal Santulli stoma refers to the end-to-side anastomosis of the distal and proximal intestinal tubes, and then, the proximal intestinal tube is pulled out of the abdominal wall to fix the fistula [12]. It can maintain the continuity of the intestinal canal and increase the absorption of nutrients and water and also make fistula closure surgery easier and faster [13]. Santulli stoma is widely used in NEC and intestinal atresia [14], but there is no report on the surgical application of IND. In recent years, Santulli stoma has been applied in our department to treat IND with good clinical effect. The novelty and purpose of this study are aimed at comparing the clinical efficacy of Santulli stoma and double-lumen stoma on IND for the first time.

## 2. Patients and Methods

### 2.1. Patients

This study was based on a retrospective controlled study conducted at a Children's Central Hospital in Fujian Province, China. This study included patients who underwent fistula surgery in our hospital due to low intestinal obstruction from January 2014 to January 2019, these children were pathologically diagnosed as IND and all underwent fistula closure surgery in our hospital, and the indications for the first operation were all the same. After admission, the symptoms of these patients could not be alleviated after conservative treatment such as gastrointestinal decompression with fluid replenishment, glycerine enema, purging, and bowel cleansing, so an exploratory laparotomy is needed. After the fistula, vomiting and abdominal distention were relieved, and normal eating was allowed. After 3-12 months, secondary closure fistula was selected for all patients, and distal fistula bowel resection was not required for all patients, as shown in Figure 1. A preprint has been published [19].

### 2.2. Inclusion and Exclusion Criteria

Inclusion criteria: (1) all patients meet the diagnostic criteria of IND: more than 20% giant ganglia in the submucosa, with more than eight neurons each on 25 ganglia, and children aged over 1 year. (2) All patients presented with severe progressive abdominal distention, vomiting, malnutrition, and less defecation on admission; vertical radiographs of the abdomen indicated low-level incomplete ileus. (3) The children were treated for abdominal distention and constipation at an age of less than 1 month. (4) Ileal double-lumen stoma or Santulli ileum stoma was performed, and fistula closure was completed in our hospital. (5) The postoperative pathological diagnosis was confirmed as congenital intestinal neuronal dysplasia (IND).

Exclusion: congenital Hirschsprung's disease and other types of Hirschsprung's homology; anorectal malformation; accompanied by other serious organic diseases and loss of follow-up.

### 2.3. Observational Indicators

The weight of children before secondary fistula closure, the time between two surgeries, the number of hospitalizations due to enteritis and dehydration between two surgeries, and the expenses related to fistula between two surgeries were collected and compared between the two groups.

### 2.4. Statistical Methods

SPSS 19.0 software was used for statistical analysis. Quantitative data were expressed as mean standard deviation, and independent sample *t*-test was used for statistical analysis. Qualitative data were compared between groups by the chi-square test. *P* < 0.05 was considered statistically significant.

## 3. Result

A total of 23 cases (12 males and 11 females) were included in this study, among which 10 cases underwent ileal Santulli stoma surgery (Santulli group) and 13 cases underwent double-lumen ileum fistula (double barrel group). There were no significant differences in baseline data (including gender, preoperative age, and weight) and stoma location between the two groups. Compared with the double-lumen group, the Santulli group had significantly higher weight of fistula precursor (*P* < 0.05), the interval between two operations was shorter (*P* < 0.05), there is less hospitalization for enteritis and dehydration during the two operations (*P* < 0.05), and there is less economic cost after fistula (*P* < 0.05); you can see Tables 1 and 2 for details.

## 4. Discussion

Allied Hirschsprung's disorder (HAD) is a general term for a group of diseases in which intestinal ganglion cells are present but their number or function is abnormal. In the neonatal period, it often causes unexplained intestinal obstruction and even intestinal perforation, requiring emergency surgery. During the operation, there is no obvious appearance of Hirschsprung's colon, such as the stenosis segment, the transitional segment, and the expansion segment, and some of them are characterized by uniform colon stenosis with intestinal wall hyperemia and edema or thick and stiff intestinal wall [3]. Intraoperative frozen rapid section can only determine the presence or absence of ganglion cells and is not yet able to make an accurate diagnosis of complex neuropathy such as abnormal development of intestinal neurons. Multisite full-thickness colorectal biopsy is a reliable means to confirm HAD [4–6]. As an important part of HAD, intestinal neuronal dysplasia (IND) has its own unique pathological characteristics [15]. Ganglion cells often exist in the intestinal nervous system, but there are abnormal changes, with the increase of ganglion cells in the unit nerve cluster and the occurrence of giant ganglion [16]. If some children with intestinal neuronal dysplasia do not have severe intestinal obstruction, conservative treatment can be performed, and surgical treatment can only be considered if conservative treatment fails [17]. However, ileostomy is a relatively feasible surgical method for children with the onset and rapid development of the disease in the neonatal period [18]. It has been reported that double-lumen fistula is often performed [19], while our department has carried out ileal Santulli fistula in recent years. From the statistical results of this study, it can be seen that there are significant differences in postoperative recovery of children by the two colostomy methods.

After double-lumen ileum fistula, only the small intestine is left to absorb nutrients, and there is no ileocecal part. Therefore, the excretion through the fistula is generally loose stools with a large amount of defecation, resulting in nutritional absorption inferior to normal children of the same age [20]. However, after Santulli fistula, in addition to defecation at the stoma, some intestinal contents can continue to be transmitted distally to the anus for excretion, increasing nutrient absorption in this part [13, 21]. In addition, if the distal defecation volume gradually increases after the fistula, the fistula can be partially or completely blocked, thus further increasing the amount of nutrition absorbed by the whole gastrointestinal tract. Therefore, the results of this study showed that the body weight of children undergoing Santulli fistula was significantly better than that of children undergoing double-lumen fistula during the second operation.

Because ileostomy basically drains loose stools, when children develop diarrhea and dehydration due to intestinal infection, it is easy to lead to severe water and electrolyte disorders and often requires emergency infusion treatment in hospital. But after Santulli fistula, we can partially or completely block the stoma, increase the nutrient absorption of the whole gastrointestinal tract, and greatly improve the absorption of water and electrolyte [22]. Therefore, children are not prone to severe dehydration due to enteritis and diarrhea. In this study, it was found that dehydration after Santulli fistula was significantly improved compared with that after double-lumen ileum fistula.

When to perform secondary closure fistula after fistula mainly depends on two conditions: (1) whether the function of the distal intestinal canal of the colostomy is restored and (2) what is the nutritional status of the second-stage operation. Recovery of intestinal function requires continuous injection of stool into the lumen to stimulate the development of intestinal ganglion cells. After double-cavity fistula surgery, doctors often need to teach family members to take stool from the proximal fistula and inject it into bowel cavity from the distal fistula anteriorly or retrograde from the anus to bowel cavity. However, neither method can guarantee that all stool can easily and completely pass through the distal intestinal canal of the ostomy. This kind of operation is complicated, and children are also more difficult to bear it. After Santulli fistula, the proximal stool can be diverted into the distal intestine only by sealing the fistula with silicone balloon catheter. The function of the distal bowel was determined by abdominal distention and anal defecation. If the abdomen is distended and defecation from the anus is not enough after sealing, the filled volume of the balloon can be reduced so that part of the stool is discharged from the fistula again. By adjusting the size of the balloon, the volume of stool passing through the distal intestinal canal of the stoma can be controlled. Therefore, Santulli stoma can better stimulate the development of the distal intestinal canal and judge whether the function of the distal intestinal canal is well recovered earlier. In this study, we found that children with Santulli fistula had a shorter interval between two operations.

In this study, it was also found that the economic cost of homecare after Santulli fistula was significantly lower than that of double-lumen fistula. Through communication with the family members, we learned that since the stool was partially discharged from the anus, the amount of stool at the fistula mouth was less than that after the double-cavity fistula operation, and the nutrition absorption was significantly improved, so there was no need to increase the amount of food intake. After sealing the fistula, the number of fistula bags used was also significantly reduced. At the same time, these children were also less likely to require multiple hospitalizations due to severe diarrhea and dehydration, and doctors were able to start secondary surgery earlier. Therefore, the total treatment cost of Santulli fistula is significantly less than that of double-lumen fistula. Ileal Santulli fistula is more recommended for infants with emergency surgery due to intestinal neuronal dysplasia, which has many advantages without obvious defects and is worth promoting.

## 5. Conclusion

For children with dysplasia of intestinal neurons, the clinical effect of ileal Santulli fistula is significantly better than double-lumen ileal fistula, which is not only beneficial to the growth and development of children after their first fistula but also shortens the time of fistula closure, reduces the incidence of dehydration, and alleviates the economic burden of their families. Therefore, it is worthy of clinical promotion and application. However, this study was only a single-center case study, which requires the participation of more children central hospitals and more cases for further verification.

## Figures and Tables

**Figure 1:** Diagram of fistula surgery.

**Table 1:** General baseline information and fistula location of the children.

	Case number	Sexuality		Age (day)	Weight (gram)	The distance between stoma and Treitz's ligament (cm)
		Male	Female			
Ileal Santulli stoma	10	5 (50.0)	5 (50.0)	29.0 ± 2.58	3807.0 ± 249.20	89.9 ± 3.54
Double-lumen ileum fistula	13	7 (53.8)	6 (46.2)	30.2 ± 3.42	3852.0 ± 235.70	90.6 ± 3.89
*t*/*χ*_2_		0.0335		-0.79	-0.376	-0.493
*P*		0.854		0.45	0.715	0.633

**Table 2:** Comparison of results between the two groups of cases.

	Body weight (g)	Postoperative cost (yuan)	Time between two operations (days)	Number of hospitalizations due to dehydration
Ileal Santulli stoma	6003.0 ± 209.39	4524.0 ± 286.33	82.0 ± 4.54	1 (10.0)
Double barrel group	4959.0 ± 171.43	7118.0 ± 489.83	103.6 ± 5.72	3 (23.1)
*t*	14.239	-13.679	-11.04	-2.449
*P*	<0.001	<0.001	<0.001	0.037

## Data Availability

The labeled dataset used to support the findings of this study is available from the corresponding author upon request.
